The article "Advances in Heavy Metal Bioremediation: An Overview" was retracted in 2023. Reasons: signs of a paper mill; compromised peer review; unreliable results or conclusions.

# Advances in Heavy Metal Bioremediation: An Overview

**DOI:** 10.1155/2021/1609149

**Published:** 2021-11-11

**Authors:** Ali Sayqal, Omar B. Ahmed

**Affiliations:** ^1^Chemistry Department, Faculty of Applied Science, Umm Al-Qura University, Makkah, Saudi Arabia; ^2^Department of Environmental and Health Research, The Custodian of the Two Holy Mosques Institute of Hajj and Umrah Research, Umm Al-Qura University, Makkah, Saudi Arabia

## Abstract

The pollution of toxic heavy metals is considered one of the most important environmental issues which has accelerated dramatically due to changing industrial activities. This review focuses on the most common methods, strategies, and biological approaches of heavy metal bioremediation. Also, it provides a general overview of the role of microorganisms in the bioremediation of heavy metals in polluted environments. Advanced methods of heavy metal remediation include physicochemical and biological methods; the latter can be further classified into in situ and ex situ bioremediation. The in situ process includes bioventing, biosparging, biostimulation, bioaugmentation, and phytoremediation. Ex situ bioremediation includes land farming, composting, biopiles, and bioreactors. Bioremediation uses naturally occurring microorganisms such as *Pseudomonas*, *Sphingomonas*, *Rhodococcus*, *Alcaligenes*, and *Mycobacterium*. Generally, bioremediation is of very less effort, less labor intensive, cheap, ecofriendly, sustainable, and relatively easy to implement. Most of the disadvantages of bioremediation relate to the slowness and time-consumption; furthermore, the products of biodegradation sometimes become more toxic than the original compound. The performance evaluation of bioremediation might be difficult as it has no acceptable endpoint. There is a need for further studies to develop bioremediation technologies in order to find more biological solutions for bioremediation of heavy metal contamination from different environmental systems.

## 1. Introduction

Heavy metals refer to metals with relatively high densities (more than 5gm/cm^3^), atomic weights (greater than 50), and atomic numbers. They are often present in the earth as a normal component due to erosion process to rocks, naturally occurring decay of plant and animal waste matter, precipitation or atmospheric accumulation of airborne particles from volcanic eruption, and forest fire smoke. Moreover, wind erosion and oceanic spray also contribute to the exposure of heavy metals in the environment [1]. The pollution of toxic heavy metals is considered one of the most important environmental issues that has been accelerated dramatically due to changing industrial activities. Pollutants can be introduced and built up in the environment due to various human activities such as domestic waste, vehicles emission, industrial processes (e.g., electroplating, dyeing, and mining), the random disposal of electronic waste, agricultural fields, sewage sludge, and waste treatment plants [2, 3]. In addition, heavy metals may be present at high levels in aquatic and soil ecosystems as compared with the atmosphere (e.g., vapors or particulate) [4, 5]. The source of heavy metals may be either natural or due to human activities, which eventually leads to their presence in soil, water, and air [5–8] (Figure 1). Contaminated soils and ground waters put human health at risk through the consumption of food grown on polluted areas, dermal contact, and the inhalation of dust [9–11]. Pollution by heavy metals is a serious threat to environmental living organisms depending on the concentration of heavy metal and the overdose absorbance rate. The negative impact of heavy metals to human and animal health is related to their long-term presence in the environment, and many heavy metals have high level of toxicity even at low concentrations (e.g., mercury, arsenic, lead, fluorine, and cadmium) [12–14]. Lead is considered one of the most persistent heavy metals because it can persist in soil up to 5,000 years with a high average biological half-life [15]. The main problem with heavy metals is the difficulty of biodegradation when bioaccumulation occurs in tissues. They are also capable of biomagnification along with the nutritional levels [16]. The discharge of heavy metals in the environment occurs through geological process (e.g., weathering and volcanic eruptions). Arsenic, lead, cadmium, nickel, chromium, cobalt, zinc, and selenium are highly toxic even in minor concentrations [17, 18]. Remediation can be defined as the removal of pollution or contaminants from the environment (e.g., sediment, groundwater, and surface water and soil) to protect human health and restore the environment. This review discusses advances in heavy metal bioremediation from the existing literature by collecting databases and information from more than 60 publications that address the last issues related to bioremediation in the context of polluted environments. It also focuses on the most common methods, strategies, and biological approaches of heavy metal bioremediation and provides a general overview of the role of microorganisms in the bioremediation of heavy metals in polluted environments.

## 2. Methods of Heavy Metal Remediation

In recent years, variable technologies and methods have been used in heavy metal remediation in contaminated environments such as soil and water. Such methods include physicochemical and biological methods; the latter is further classified into in situ and ex situ bioremediation.

### 2.1. Physicochemical Methods

Physicochemical methods include processes that work to remove heavy metals from any contaminated environment. They can be applied on the form of particulate of metals or metal-containing particles. This remediation can be conducted through physical and chemical processes such as ion exchange, precipitation, reverse osmosis, evaporative recovery, solvent extraction, filtration, chemical oxidation, chemical leaching, electrokinetics, land filling, electrochemical treatment, electrodialysis, ultrafiltration, solvent extraction, chemical precipitation, chemical reduction, and isolation (mechanical) separation of metals [1, 9, 19, 20]. However, these methods may show incomplete metal removal; in addition, they require high solvent and production of poisonous waste products. They also have an inherent negative environmental impact and are usually soil disturbing, besides that fact that they are labor intensive and expensive [10]. So, these methods are limited by their high costs, high energy requirements, low efficiency, unpredictable metal ion removal, and generation of toxic sludge [21–27].

### 2.2. Biological Methods

Biological remediation or biodegradation constitutes many types of methods involved in the removal or degradation of heavy metals through biological activity. These biological treatments may either include aerobic (presence of oxygen) or anaerobic (absence of oxygen) processes and can be used for heavy metal removal. Biodegradation is a process wherein the polluted environment is biologically degraded under certain conditions to levels below the concentration limits established by regulatory authorities [28–32]. Bioremediation can further be classified into in situ or ex situ categories based on the strategies involved in Table 1.

#### 2.2.1. In Situ Bioremediation

In situ bioremediation methods treat the contamination at the site without removing soil. The use of these specific methods depends on many factors: the area contaminated, properties of the compounds involved, concentration of the contaminants, and time required to complete the bioremediation. This process is usually recommended because it requires moving fewer materials and is less expensive. In situ bioremediation is sometimes classified into intrinsic bioremediation and engineered in situ bioremediation. It includes so many types mainly bioventing, biosparging, biostimulation, bioaugmentation, and phytoremediation [33–36].

*(1) Bioventing*. Bioventing technique is the most commonly used in situ mechanism in which air and nutrients are supplied to polluted soil to stimulate the microorganisms (bacteria). Bioventing requires limited air flow and low oxygen rates to release pollutants to the atmosphere through biodegradation. It can simulate in situ biodegradation of simple hydrocarbons in the soil, and hence, the contamination occurs deep under the surface [37]. Bioventing is limited by the inability to deliver oxygen to the polluted soil and the insufficient aeration of shallow contamination [38].

*(2) Biosparging*. Biosparging is defined as the injection of law pressure air below the water table to raise the level of groundwater oxygen and enhance the rate of bacterial bioremediation of contaminants [33]. Both bioventing and biosparging techniques have been utilized simultaneously to guarantee the efficient removal of the soil contaminants despite any unfavorable conditions. Biosparging can also combine soil and groundwater to reduce the concentration of dissolved oil compounds in groundwater, mixed with soil under level under water table and within the capillary fringe. It is an ease and low-cost procedure with considerable flexibility.

*(3) Biostimulation*. Biostimulation involves enhancing bacterial growth to initiate the bioremediation process. First, the polluted soil is mixed with enriched nutrients and vital substances to stimulate microbial activity for the fast degrading of contaminants or toxic compounds into the carbon source or nitrogen and phosphorous source [39]. Microorganisms such as bacteria and fungi represent nature's original recyclers. The capability of microorganism to transform chemical pollution into sources of energy and useful materials suggests important biological processes which are lower in cost and friend to environment.

*(4) Bioaugmentation*. In bioaugmentation, there are certain sites where microorganisms are required to extract the contaminants. They are also able to outcompete indigenous microorganisms, which means that they can clean up the site rapidly. The removal of toxic chemicals through bioaugmentation has been reported in environments such as soil and water. However, a number of limitations have also been documented. For instance, it has been observed that there is a decrease in the number of exogenous microorganisms after their addition to a polluted site due to abiotic and biotic stresses. They occur due to insufficient growth nutrients such as substrates, temperature changes, and pH, in addition to the competition between introduced and indigenous microorganisms [40, 41].

*(5) Phytoremediation*. Phytoremediation represents an emerging technology that uses plants to remove pollution from soil and water. It has a potential use in the biodegradation of organic contaminants and may be a promising choice in the future. This technology is suitable for sites with shallow contaminants. Nevertheless, many studies have highlighted several limitations of this technology, such as contamination concentration, toxicity, bioavailability, the type of plant, and stress tolerance [42].

#### 2.2.2. Ex Situ Bioremediation

Ex situ bioremediation means excavating and treating soil prior to returning the soil to its original state. If the contaminated material is excavated, it can be treated on or off site, which is often a more rapid method of decontaminating the area. Ex situ bioremediation is categorized into solid phase and slurry phase systems. The most important techniques include land farming, composting, biopiles, and bioreactors [33].

*(1) Land Farming*. Land farming is a simple process which implies that excavation of contaminated soil over a prepared site with periodic tilling until pollutants is degraded through microorganisms where the practice is limited to the treatment of small part of soil [43]. The technique is easy and much effective specially when used for petroleum-contaminated soil. However, the technique is limited to the treatment of a small space of upper soil (10–35 cm).

*(2) Composting*. A composting method involves combining polluted soil with nonhazardous organic agricultural wastes to support the growth of high microbial number with increased temperatures (40-65°C). The method is applied to a mixture of excavated soils and biosolids (wood chips, animal, and vegetative wastes) contaminated with organic materials (petroleum hydrocarbons and pesticides) [33, 43].

*(3) Biopiles*. Biopiles are a mix or hybrid between land farming and composting. Biopiles produce enriched environments for different microorganisms (both aerobic and anaerobic). The aqueous reactors represent an ex situ treatment of a contaminated environment, where reactors are pumped up from a certain site. It involves bioremediating a contaminated environment by using a special engineered technology [33]. Engineered cells are made for the treatment of surface pollutants to regulate physical losses of the contaminants through leaching, which is then followed by volatilization [43]. Biopiling is considered a feasible, cost-effective technique for contaminated soils.

*(4) Bioreactor*. A bioreactor is a vessel used after a certain optimization of an external environment in which a biochemical reaction occurs. The system may include enzymes, tissues, microorganisms, and animal and plant cells to achieve a high yield of bioremediation. Overall, biodegradation is higher in bioreactor systems as compared with other systems because the target environment is easy to manage, control, and predict. Despite the advantages of reactor systems, it is found that the contaminated environment (e.g., soil) requires excavation of the contaminant from the soil through physical extraction before being processed by a bioreactor [33].

## 3. Role of Microorganisms

Various species of microorganisms can be used for bioremediation, as they are nature's original recyclers. They are also capable of transforming chemicals into sources of energy and raw materials for their own growth to produce a low-cost and environment-friendly biological process. Due to their high industrial use, heavy metals have become a worldwide real environmental problem. Toxic heavy metals are accumulated through the food chain due the industrial activities and fuel consumption leading to both environmental and health problems. These heavy metals exert toxic effects on living cells (mercury, silver, lead, cadmium, and arsenic). Many types of bacteria carry resistant genes to many types of cations and oxyanions of heavy metals in their DNA. To survive, bacteria undergo many different mechanisms to face the uptake of heavy metal ions. These mechanisms include biosorption, entrapment, efflux, reduction, precipitation, and complexation. Microorganisms therefore can be a promising, unlimited resource for new environmental biotechnologies. Bioremediation uses naturally occurring microorganisms to degrade or detoxify hazardous substances to human health and/or the environment. The microorganisms can either be used indigenously or be isolated from other resources at the polluted site [44, 45]. Microorganisms which are involved in biodegradation are shown in Table 2, including the following examples: *Acinetobacter*, *Actinobactera*, *Alcaligenes*, *Arthrobacter*, *Bacillins*, *Beijerinckia*, *Flavobacterium*, *Methylosinus*, *Mycobacterium*, *Mycococcus*, *Nitrosomonas*, *Nocardia*, *Xanthobacter*, *Penicillium*, *Phanerochaete*, *Pseudomonas*, *Rhizoctonia*, *Trametes*, and *Serratia* [46–66]. Most bioremediation processes are completed under aerobic conditions, but running a system under anaerobic conditions may permit microbial organisms to degrade otherwise recalcitrant molecules [44]. Aerobic organisms depend on oxygen during their growth activity. These are continuous processes which are known as cellular respiration, which use oxygen to oxidize substrates like fatty acid from oil in order to obtain energy. Examples of degradative aerobic bacteria are *Pseudomonas*, *Sphingomonas*, *Rhodococcus*, *Alcaligenes*, and *Mycobacterium*. Microorganisms can also be used to degrade toxic chemicals such as pesticides besides hydrocarbons materials [33]. Many bacteria use the contaminant as a metabolic source (carbon and energy). An anaerobic bacterium is an organism that does not need oxygen as a based metabolism, and it differs from aerobic bacteria. Anaerobic bacteria have also been used for the bioremediation of biphenyls, dechlorination, and chloroform [33]. Furthermore, fungi may be able to degrade a high range of persistent or toxic environmental pollutants [45]. There are many types of substrates available, such as corn cobs, straw, and dust. The aerobic bacteria that grow by utilizing methane for carbon and energy. This aerobic degradation being initiated with enzyme methane monooxygenase will be active against a wide range of chemicals [33].

## 4. Factors Affecting Bioremediation

The removal of heavy metals through microorganisms may have ecological and economic limits. Several factors should be considered for the selection of a proper bioremediation. There are certain variables that have a great impact on the extent of biodegradation. First, nutrients in the polluted environment such as nitrogen, phosphate, sulphur iron, and potassium can stimulate and support strong microbial growth, cellular metabolism, and microorganism growth [34]. These nutrients represent basic life requirements and help microorganisms produce necessary enzymes to break down contaminants. Second, the remediation cost may also play an important role in the continuity of bioremediation, meaning that the cost should be low for financial feasibility. Third, the nature of pollutants, meaning whether they are solid, semisolid, liquid, or volatile in nature, may affect the process, or the pollutants are toxic or nontoxic, organic, and inorganic pollutants, heavy metals, polycyclic aromatic hydrocarbons, pesticides, and chlorinated solvents. The nature of the polluted area is also highly important, as it can affect the quality of bioremediation. Fourth, pH, temperature, and other physicochemical factors are important for the bioremediation process. The selection of the optimum range of these parameters can also greatly influence the rate and extent of biodegradation, as it influences the microbial growth and hence the removal of the contaminants [33]. Fifth, moisture content (water) is also a primary factor for biological growth and efficient bioremediation. Sixth, microbial diversity that can biodegrade any contaminant such as Pseudomonas, Aeromonas, Flavobacteria, Aeromonas, Chlorobacteria, Corynebacteria, Acinetobacter, Mycobacteria, Streptomyces, Bacilli, Macrobenthos, and other aquatic plants such as E. crassipes and L. hoffmeisteri can also degrade turbidity and chemical domestic wastewater [35]. Seventh, oxygen is mainly used for the initial breakdown of the hydrocarbon in the contaminated sites and also can be used for both aerobic and anaerobic bioremediation [36].

## 5. Advantages and Limitations

Bioremediation is a simple process used by many scientists in the waste treatment process for contaminated environments such as soil. The microbes that degrade the contaminant increase in numbers and release harmless products. The residues for the treatment are usually harmless products such as carbon dioxide, water, and cell biomass. Bioremediation is of very less effort, less labor intensive, and cheap compared to other methods that are used for the removal of hazardous waste. Bioremediation is also ecofriendly, sustainable, and relatively easy to implement. It is also useful for the complete destruction of a wide variety of contaminants [64]. Many hazardous compounds can be transformed into harmless products. Moreover, bioremediation can be implemented on the site of contamination itself without causing a major disruption of normal activities. There is no need to transport large numbers of waste off-site, there is no potential human health risk, and the environment will remain uncontaminated. Most of the disadvantages of bioremediation relate to it needing a longer time to be completed as compared with other options such as excavation and removing pollutants from the site. Also, there is a difficulty of bioremediation in treating inorganic contaminants and in confirming whether contaminants have been destroyed or not. Besides that, there is a slowness of highly chlorinated materials biodegradation and generation of more toxic or carcinogenic by-products [65, 66]. Furthermore, the products of biodegradation sometimes become more toxic than the original compound. Its biological processes are also highly specific. Examples for effective site factors include the presence of microbial populations, growth conditions, and quantity of nutrients and pollutants [33, 65].

## 6. Conclusion

Bioremediation technique is still a useful, natural, and environmentally friendly process in which the polluted environment is biologically biodegraded. Microorganisms play a significant role in the removal of heavy metals pollutants. The heavy metals (e.g., mercury, silver, lead, cadmium, and arsenic) exert toxic effects on living cells. Examples of degradative aerobic bacteria are *Pseudomonas*, *Alcaligenes*, *Sphingomonas*, *Rhodococcus*, and *Mycobacterium*. Anaerobic bacteria have also been used for the bioremediation of biphenyls, dechlorination, and chloroform. Furthermore, fungus microorganisms can effectively degrade many toxic environmental pollutants. Phytoremediation represents an emerging technology through which plants can be used to remove pollution from soil, water, and other environments. Bioremediation is of very less effort, less labor intensive, cheap, ecofriendly, sustainable, and relatively easy to implement. Most of the disadvantages of bioremediation relate to the slowness and time-consumption; furthermore, the products of biodegradation sometimes become more toxic than the original compound. Bioremediation may be limited by irregularity and uncertainty of completeness. Also, the performance evaluation of bioremediation might be difficult as there is no acceptable endpoint. There is a need for further studies to develop bioremediation technologies in order to find more biological solutions for bioremediation of heavy metal contamination from different environmental systems.

## Figures and Tables

**Figure 1:** Sources and cycles of heavy metals in the environment [5].

**Table 1:** Types of bioremediation.

Strategy	Degradation	Organism	References
In situ bioremediation Bioventing Biosparging Biostimulation Bioaugmentation Phytoremediation	Biotransformation	Bacterioremediation	[32–36]
Ex situ bioremediation Land farming Composting Biopiles Bioreactors	Biodegradation	Mycoremediation	
Others	Mineralization	Phytoremediation	
		Compost bioremediation	

**Table 2:** Heavy metal distribution in environment and microorganisms involved in biodegradation.

Heavy metal	Distribution	Microorganism	Reference
As	Soil, volcanic eruption	*Sporosarcina ginsengisoli*	[46, 47]
Cd	Soil, sedimentary rocks, water	*Bacillus sp.* *Klebsiella planticola*	[48–50]
Cr	All environments	*Bacillus cereus strain XMCr-6* *Bacillus cereus* *Pseudomonas putida* *Enterobacter cloacae B2-DHA* *Bacillus subtilis*	[51–54]
Pb	Soil	*Rhodobacter sphaeroides* *Leclercia adecarboxylata* *Kocuria flava*	[55]
Hg	Water, soil, and air	*Bacillus* sp. strain CSB_B078 *Klebsiella pneumoniae* isolate *Enterobacter* sp. strain 08 *Acinetobacterseohaensis* strain	[56]
Cu	Earth's crust, oceans, lakes, and rivers	*Kocuria flava*	[57]
Zn	Surface water, soil, and rock	*Pseudomonas putida*	[58, 59]
Ni	Air, soil, sediments, and water	*Desulfovibrio desulfuricans* Bacillus licheniformis	[60, 61]
Co	Air, soil, and water	*Bacillus* sp. *Rhodopseudomonas palustris*	[49, 62, 63]

As: arsenic; Cd: cadmium; Cr: chromium; Pb: lead; Hg: mercury; Cu: copper; Zn: zinc; Ni: nickel; Co: cobalt.
